The article "Amyotrophic lateral sclerosis and delayed onset muscle soreness in light of the impaired blink and stretch reflexes – watch out for Piezo2" was published in 2022. Journal: Open Med (Wars).

# Amyotrophic lateral sclerosis and delayed onset muscle soreness in light of the impaired blink and stretch reflexes – watch out for Piezo2

**DOI:** 10.1515/med-2022-0444

**Published:** 2022-03-01

**Authors:** Balázs Sonkodi, Tibor Hortobágyi

**Affiliations:** Department of Health Sciences and Sport Medicine, University of Physical Education, Budapest, Hungary; ELKH-DE Cerebrovascular and Neurodegenerative Research Group, Department of Neurology, University of Debrecen, Debrecen, Hungary; Department of Pathology, Faculty of Medicine, University of Szeged, Szeged, Hungary; Department of Old Age Psychiatry, Psychology and Neuroscience, King’s College London, London, UK; Center for Age-Related Medicine, SESAM, Stavanger University Hospital, Stavanger, Norway

**Keywords:** amyotrophic lateral sclerosis, delayed onset muscle soreness, extraocular muscle, stretch reflex, blink reflex, Piezo2 ion channel

## Abstract

Amyotrophic lateral sclerosis (ALS) is a fatal, multisystem neurodegenerative disease that causes the death of motoneurons (MNs) progressively and eventually leads to paralysis. In contrast, delayed onset muscle soreness (DOMS) is defined as delayed onset soreness, muscle stiffness, loss of force-generating capacity, reduced joint range of motion, and decreased proprioceptive function. Sensory deficits and impaired proprioception are common symptoms of both ALS and DOMS, as impairment at the proprioceptive sensory terminals in the muscle spindle is theorized to occur in both. The important clinical distinction is that extraocular muscles (EOM) are relatively spared in ALS, in contrast to limb skeletal muscles; however, the blink reflex goes through a gradual impairment in a later stage of disease progression. Noteworthy is, that, the stretch of EOM induces the blink reflex. The current authors suggest that the impairment of proprioceptive sensory nerve terminals in the EOM muscle spindles are partially responsible for lower blink reflex, beyond central origin, and implies the critical role of Piezo2 ion channels and Wnt-PIP2 signaling in this pathomechanism. The proposed microinjury of Piezo2 on muscle spindle proprioceptive terminals could provide an explanation for the painless dying-back noncontact injury mechanism theory of ALS.

## 1 Introduction

Charcot, a French neurologist, wrote about amyotrophic lateral sclerosis (ALS) first in the 19th century [1]. ALS is a fatal, multisystem neurodegenerative disease that causes the death of motoneurons (MNs) progressively [2,3]. On the other hand, Theodor Hough described delayed onset muscle soreness (DOMS) in 1902, ascribing the cause of muscle rupture [4]. However, the exact pathomechanism is far from known in ALS and the case is not different in DOMS either. DOMS is defined as delayed onset soreness, muscle stiffness, loss of force-generating capacity, reduced joint range of motion and decreased proprioceptive function [5]. The current authors emphasize the sensory deficits and impaired proprioception as common symptoms of both DOMS [5,6,7] and ALS [8,9,10]. Nevertheless, this was not the case for a long time when clinicians, for example, did not consider sensory neuronal and eye involvement as part of the features of ALS, and generally, it was considered as a pain-free lethal disease [10,11]. Emerging research studies have started to highlight the importance of sensory circuit dysfunction in ALS [10,12,13,14]. Correspondingly, both ALS and DOMS are suggested to be associated with impairment at the proprioceptive sensory terminals in the muscle spindles [7,10,15]. Furthermore, the recent ALS dying-back injury mechanism theory put forward the muscle spindle-derived sensory degeneration that induces the nonresolving progressive impairment of the proprioceptive circuitry [10].

The article "Amyotrophic lateral sclerosis and delayed onset muscle soreness in light of the impaired blink and stretch reflexes – watch out for Piezo2" was published in 2022. Journal: Open Med (Wars).

The important clinical distinction is that extraocular muscles (EOM) are spared from progressive degeneration in ALS, in contrast to limb skeletal muscles [1,16,17,18]. The question has been on the agenda, why? Furthermore, the stretch of EOM is suggested to induce blink reflex [19]. However, the blink reflex goes through impairment in the later stage of ALS, regardless of relatively spared EOM. Moreover, a new DOMS hypothesis implies that the primary cause of this noncontact injury is a transient mechano-energetic impairment of the Piezo2 ion channel on the proprioceptive terminal of the muscle spindles, leading to a significant delay in the medium latency response of the stretch reflex (MLR) [10,15]. The question that arises is whether there is a mechanistic link between the aforementioned and with the delayed latency of {\text{R}}_{2}^{^{\prime} }] , R_2_ and R_1_ components of the blink reflex? By answering these questions, we could possibly reveal further the difference in this distinct preservation phenomenon and could provide additional clues in reference to the degeneration mechanism of ALS.

## 2 Blink reflex, extraocular muscle spindle, and proprioception

Blink is a burst bilateral eyelid closure associated with concomitant eye movements. It provides a protective barrier for the eyes and facilitates the distribution of the tear film on the corneal surface. Accordingly, harsher tapping of the eyes elicits a bilateral blink reflex with the features of a nociceptive reflex [19]. Blink reflex is an oligosynaptic reflex comprising three neurons and transduced by the trigeminal and facial nerves [11]. The short-latency blink reflex is induced by the stretching of EOM and elicited in the EOM muscle spindles [19]. Muscle spindles contribute to the stretch reflex, and electromyographic studies clearly demonstrated stretch reflex responses in EOM of humans [20,21,22,23].

The article "Amyotrophic lateral sclerosis and delayed onset muscle soreness in light of the impaired blink and stretch reflexes – watch out for Piezo2" was published in 2022. Journal: Open Med (Wars).

There are six EOM controlling eye muscles. The motor units of EOM are distinguished from other muscles because they have a special set of myosin heavy chains and they also have multiple neuromuscular innervation sites per single myofiber [24]. An interesting hallmark of ALS is that EOM enjoy a relative resistance to this lethal disease even until the later stage of progression, in contrast to skeletal muscles of extremities [1,16,17,18].

Our knowledge about the MNs of EOM is fairly well-founded, in contrast to our knowledge pertaining to the sensory innervation of EOM [25]. Muscle spindles and myotendinous cylinders (palisade endings) are the two types of sensory receptors located in EOM [25]. Noteworthy is, that, the structure of EOM muscle spindles differs from the ones found in skeletal muscles [25,26]. Since the density of EOM muscles spindles is comparable to the one found in hand and neck muscles, it leads to the suggestion that they have a role in fine motor control and possibly in proprioception [25]. Excitation of the EOM afferents could be detected in higher brain regions [25].

## 3 Microinjury of the Piezo2 ion channel in proprioceptive terminals

A recent hypothesis in reference to the cause of DOMS concludes that the primary injury of this dichotomous noncontact injury is a transient microdamage of the Piezo2 ion channel at the proprioceptive terminal in the muscle spindle [7,15]. Piezo proteins are enormous channels in size and with several transmembrane segments [27]. Yet, our knowledge pertaining to their topology, pore formation, mechanical force detection, and gating mechanism is substantially limited [27]. Noteworthy is, that, Piezo2 was found to be the principal transduction channel for proprioception [28]. Important underlying factors that could lead to the proposed acute Piezo2 channelopathy in DOMS are repetitive lengthening contractions leading to proprioceptive hyperexcitation, fatigue, and eventually, cognitive demand induced acute stress reaction (ASR) [7,15]. Note that these factors are implicated in the dying-back noncontact injury mechanism of ALS as well [10].

The suggested transient Piezo2 channelopathy mechanism in DOMS is as follows. The peripheral ending of proprioceptive nerves in the muscle spindle is theorized to be exposed to a terminal arbor degeneration (TAD)-like lesion [7], as could be observed as a side effect of platinum-analogue chemotherapy [29]. Bennett et al. wrote about TAD as, “if the energy deficiency is severe enough then degeneration happens, and the threshold for degeneration will be lowest in the neuronal compartment that has the highest energy requirement” [29] and that could be the axon terminals of hyperexcited proprioceptive nerves [7,10]. Accordingly, the peripheral endings of the proprioceptive sensory neurons in the muscle spindle are densely populated with mitochondria [30]. Cognitive demand-derived ASR induces mitochondrial energy depletion on top of unaccustomed or strenuous repetitive eccentric contractions, meaning hyperexcited proprioceptive fibers could guide the way toward a TAD-like lesion. In due course, it turns into a pathological process and that is the microinjury of the Piezo2 ion channel. Note that the hyperexcitation-related inactivation of Piezo2 ion channels is a physiological mechanism, and therefore, it is considered to be within homeostasis [31,32]. However, the proposed microinjury is beyond this point. Correspondingly, the stress-related microinjury of Piezo2 ion channels could be translated as breaching the homeostatic limits of an overreaching response. Indeed, stress-derived modified kinetics of Piezo exists in pathology [32]. The result of this transient channelopathy is that pathological changes could occur on the other central endings of the pseudounipolar primary afferents as well [33]. The gate controllers of these pathological changes are suggested to be the activated NMDARs [10]. Correspondingly, Bewick et al. put forward earlier that glutamate was released from synaptic-like vesicles in the proprioceptive terminals of the muscle spindles in a stretch-modulated manner [34]. However, Than et al. confirmed recently that glutamate release is in fact vesicular [31,35]. Sonkodi et al. further theorized that stress-induced mitochondrial energy deficiency could impair glutamate vesicular release and that could lead the way to glutamate spillover at the primary afferent terminals [15]. In addition, they hypothesized that mechano-energetically impaired Piezo2 channels could become permeable to Piezo currents and even to glutamate when they should not [15]. Finally, glutamate excitotoxicity could activate NMDARs at presynaptic central terminals at the spinal dorsal horn with potential long-term consequences [10,15]. This microinjury mechanism could provide the base for the acute noncontact injury mechanism of DOMS and degenerating dying-back noncontact injury mechanism of ALS [7,10].

The article "Amyotrophic lateral sclerosis and delayed onset muscle soreness in light of the impaired blink and stretch reflexes – watch out for Piezo2" was published in 2022. Journal: Open Med (Wars).

Furthermore, this stress-related Piezo2 microinjury at the proprioceptive terminals is suggested to compromise the static encoding of the stretch reflex [10,15,36]. As a result, it is proposed that the impaired static encoding of the primary afferents in the muscle spindle is diverted to a secondary preprogrammed compensatory microcircuit further involving the secondary afferents and more synaptic connections [10,15].

## 4 Lower blink rate in ALS

It has been observed that familial ALS patients had significantly reduced blink rates than sporadic ALS patients and controls [11]. Even earlier it was found that the blink reflex was abnormal in both primary lateral sclerosis (PLS) and ALS [37]. It is unanswered whether the lower blink rate in ALS has a peripheral or central origin [11]. Blinking is transduced by trigeminal and facial nerves by a well-explored three-neural reflex arc [11]. Byrne et al. excluded the motoneuronal origin of the lower blink rate in ALS because the impairment of it would be associated with slower blinks instead of a lower blink rate [11]. Furthermore, they ruled out sensory neural origin based on an earlier clinical view that these nerves are not involved in the ALS pathology [11]. Finally, they proposed that a lower blink rate in familial ALS is central in origin and is probably associated with alteration in the control of spontaneous blinks [11].

Longitudinal follow-up data showed that blink reflex impairments progressed over time in ALS patients, namely, the latencies of R_2_ and {\text{R}}_{2}^{^{\prime} }] were delayed, leading to the disappearance of these components at the very late stage of ALS [37]. It has been long known that the blink reflex has two superimposed R_2_ subcomponents and R_2_ is more prone to inhibitory effects of repetitive stimulation and prepulses [38]. The dissection of R_2_ subcomponents is often challenging due to temporal overlap [38]. The gradual disappearance started at a late stage of ALS with the {\text{R}}_{2}^{^{\prime} }] subcomponent, followed by R_2_ and R_1_ and eventually there was no detectable blink reflex [37]. The alteration of the R_2_ subcomponent is devoted to the direct impairment of the stretch pathway or to other indirect lesions affecting the excitability of the reflex [39]. However, if we factor in sensory contribution, then it might lead us to a different interpretation of the above conclusions, especially in light of the new theory of DOMS [7,10,15].

Note that the electromyogram (EMG) of stretch reflex comprises three components: short latency (largely Type Ia afferent mediated), medium latency (largely dominantly Type II afferent mediated) and long-latency (probably transcortical or subcortical) responses [40,41,42,43,44,45,46,47,48,49]. It is important to note that DOMS is suggested to delay the latency of MLR of the stretch reflex [10,15]. Indeed, the recent (unpublished observations) of Sonkodi et al. supported this hypothesis. Earlier findings demonstrated that DOMS do not alter the latency of SLR and LLR [50], as the (unpublished observations) of Sonkodi et al. also found unaltered LLR. They presumed that the delayed latency of MLR is due to the minor alteration of the static encoding of the stretch reflex when monosynaptic Type Ia static proprioceptive encoding is altered to polysynaptic Type II static encoding due to the microdamage of the Piezo2 ion channels at the primary afferent endings in the muscle spindle [10,15]. On the contrary, the dynamic encoding component of the stretch reflex is hardly affected, like in the case of Oxaliplatin-based chemotherapy [51], and as a consequence, the SLR remains unaffected [10,15].

The article "Amyotrophic lateral sclerosis and delayed onset muscle soreness in light of the impaired blink and stretch reflexes – watch out for Piezo2" was published in 2022. Journal: Open Med (Wars).

Accordingly, the current authors suggest that the SLR (monosynaptic) of the stretch reflex acts analogous with the R_1_ component (three-neural) of the blink reflex, MLR (polysynaptic) is analogous with the R_2_ subcomponent (polysynaptic with similar transduction time as {\text{R}}_{2}^{^{\prime} }] ) and LLR (polysynaptic with even longer transduction than MLR) is almost like the {\text{R}}_{2}^{^{\prime} }] subcomponent (polysynaptic with similar transduction time as R_2_ and minor differences in the axon length). Furthermore, the temporal overlap of R_2_ subcomponents of the blink reflex could be due to the minimal difference in the critical axon length difference in terms of transmission as opposed to the stretch reflex responses of extremities. Since the order of impairment in ALS starts with the {\text{R}}_{2}^{^{\prime} }] subcomponent, followed by R_2_ and R_1_ components of the blink reflex [37], this could be the evidence of four implications. First, there could be a dying-forward mechanism in the late stage of ALS from the central origin to the preserved periphery as was suggested by Byrne et al. [11]; however, we propose that the somatosensory nerves could be paradoxically involved even in this degeneration mechanism because the nonresolving progressive impairment of the proprioceptive circuitry from the periphery could arrive at this stage. Second, there could be a parallel dying-back mechanism at the very late stage of disease progression from impaired proprioceptive sensory neurons to MNs as was suggested by Sonkodi [10]. Third, it is proposed by the current authors that the ALS disease advancement progressively impairs the static encoding of the affected stretch reflexes, including the blink reflex. In line with these implications, EOM are selectively unaffected in ALS [1,16,17,18]. Finally, the impairment of the static encoding of a stretch reflex could also mean the intrusion of our most profound life-sustaining preprogrammed genetic encoding [15]. Correspondingly, Fernández-Trillo et al. highlighted that these Piezo2 containing neurons have different, and most likely principal, genetic signatures [52]. No wonder why Piezo2 knockout mice cannot survive after birth [27,53] due to the lack of the homeostasis maintaining the physiological function of Piezo2 ion channels [27]. Therefore, it is safe to say that any systemic direct or indirect irreversible cause that detaches and impedes the regeneration of Piezo2 containing somatosensory neuron terminals demonstrated to be incompatible with life sustainment.

The article "Amyotrophic lateral sclerosis and delayed onset muscle soreness in light of the impaired blink and stretch reflexes – watch out for Piezo2" was published in 2022. Journal: Open Med (Wars).

A recent research study demonstrated that eye blinks of Piezo2-deficient mice were lower than wild types when the blinks were elicited by von Frey filaments [52]. It is important to note on the side that TAD lesion causing platinum-analogue chemotherapy also causes the delay of the blink reflex [54]. The involvement of the Piezo2 ion channel in the blink reflex impairment is compelling in the light of the new theory of DOMS, in which the channelopathy of Piezo2 is also implicated as the critical primary TAD-like lesion in its biphasic noncontact injury mechanism [15,55]. Note that blinks could be evoked despite corneal and conjunctival anesthesia [56], suggesting from the animal model that the spinal trigeminal complex is a principal element as a spontaneous blink generator [11,57]. Earlier findings put forward that the short-latency blink reflex is induced by the stretching of the EOM, thus it could be initiated in the extraocular muscle spindles [19]. Accordingly, the blink reflex could be considered as an oligosynaptic stretch reflex. Note that the ophthalmic branch of the trigeminal nerve comprises these muscle spindle-derived primary afferents [19].

Interestingly EOM are relatively spared in ALS [1,16,17,18]. One reason could be that Wnt protein signaling is significantly lower in human limb skeletal muscles of ALS patients than in EOM [18]. Note that increased Wnt signaling stimulates the phosphatidylinositol [4,5]bis-phosphate (PIP2) formation [58], while PIP2 is known to be involved in the control of Piezo2-dependent mechanotransduction [59]. Correspondingly, the current authors suggest that the spared level of Wnt signaling could even save the primary afferent neuromuscular junctions within the muscle spindles of EOM in ALS. Note that this neuromuscular junction in the muscle spindles is proposed to be the locus minoris resistentiae in ALS and the shortage of Wnt signaling could be one explanation for the detachment of Type Ia sensory terminals from intrafusal muscle fibers in striated muscles [10,12]. However, this sparing effect on the somatosensory side could last only until the dying-forward mechanism reaches these proprioceptive nerves. The resultant somatosensory lesions, represented in delayed latency of R_2_ and later R_1_ components, could eventually initiate the dying-back mechanism propagating toward the MNs of EOM at the very last stage of ALS disease progression but it is a lengthy process, especially under elevated Wnt signaling circumstances, and therefore it could not evolve to this point.

The article "Amyotrophic lateral sclerosis and delayed onset muscle soreness in light of the impaired blink and stretch reflexes – watch out for Piezo2" was published in 2022. Journal: Open Med (Wars).

## 5 Conclusion

The current authors put forward the late involvement of somatosensory neurons in the unanswered question of whether the lower blink rate in ALS has a peripheral or central origin. At a later stage of ALS disease progression, the impairment of proprioceptive sensory nerves in the EOM muscle spindles could be partially responsible for lower blink reflex, beyond central origin. Moreover, the current authors imply the critical role of Piezo2 ion channels and Wnt-PIP2 signaling in this pathomechanism. The proposed microinjury of Piezo2 on muscle spindle proprioceptive terminals could even provide an explanation for the painless dying-back noncontact injury mechanism theory of ALS.
